# Effects of Body Posture and Different Exercise Intensity on Athletes' Limb Injury

**DOI:** 10.1155/2022/5103017

**Published:** 2022-06-28

**Authors:** Di Jin, Qian Ma

**Affiliations:** ^1^Anhui Normal University, Wuhu, Anhui 241000, China; ^2^Wannan Medical College, Wuhu, Anhui 241000, China

## Abstract

The purpose of this study was to solve the problem of the influence of body posture and different exercise intensity on athletes' limb injuries, to meet the needs of understanding athletes' injuries, and to make up for the lack of investigations on athletes' limb injuries; this also increases the chances of an athlete avoiding injury. Severe acute sports injuries of high-level gymnasts endanger the personal safety of athletes. Many movements in gymnastics are done in the air much higher than the ground, and there is no fulcrum when the athlete does the movements; this just can only maintain balance and change your body posture through your own feelings, a slight error can easily cause your head or upper body to fall down, and the fragile spine cannot withstand the strong impact of the ground, resulting in high vertebral fractures, high paraplegia, and even death. Therefore, through a survey of 126 rhythmic gymnasts who participated in the 2011 “China Art Sports Cup” China Rhythmic Gymnastics Championship, a total of 172 injuries were found in 136 gymnasts, and the injury risk analysis was carried out from the main characteristics of the injuries.

## 1. Introduction

With the continuous development of modern rhythmic gymnastics, the competition in international competitive sports is becoming increasingly fierce; in order to pursue higher, more difficult, new, and clever technical movements, special training with high intensity and large amount of exercise is carried out; the ensuing sports injuries are becoming more and more serious, which restricts the further improvement of the athletes' competitive level. How to solve the problem of prevention, treatment, and rehabilitation of athletes' injuries, so as to ensure the normal training and competition of athletes, is an important part of competitive work [1]. Competition is usually accompanied by risks. Under the traditional thinking concept of risk “entity” school, the general understanding of risk composition is as follows: risk is composed of a variety of elements; these elements mainly refer to risk factors, risk accidents, and risk losses. They work together to determine the existence, occurrence, and development of risks [2]. Risk factors refer to conditions that are sufficient to cause or increase the possibility of a risk accident, the potential cause of a risk accident, and the inherent or indirect conditions or hidden dangers that cause losses; it promotes the occurrence of risk accidents or increases the frequency of accidents and losses. Risk events generally refer to accidental events that directly cause loss of life and property and are accidental events that directly lead to the consequences of loss, that is, the direct cause and external cause of the loss. Risk of loss is the result of unplanned, unintended, and unintentional conditions that cause economic loss or personal injury. Risk factors are the necessary conditions for the formation of risks and the premise for the occurrence and existence of risks. A risk event is a sufficient condition for the existence of a risk, central to the overall risk. Risk events are the bridge connecting risk factors and risk losses and the medium through which risks are transformed from possibility to reality. The relationship between risk factors, risk events, and risk losses can be represented by the chain of action of risk; understanding the chain of action of risk is of great significance for dealing with risks [3], as shown in Figure 1.

Risk identification is the first step in risk management; it refers to the systematic understanding and analysis of a large number of reliable information from a large number of sources, to recognize the various risk factors existing in the project, then to determine the risks faced by the project and its nature, and to grasp its development trend.

## 2. Literature Review

Skinner and Isaacs said that by conducting a trauma epidemiological study of 88 rhythmic gymnasts, research shows that the top three incidence rates of common and frequently occurring diseases in rhythmic gymnasts are chronic sacrospinalis muscle injury at 15.9%; lumbar supraspinous ligament injury, lumbar interspinous ligament injury, psoas fasciitis, and anterior talofibular ligament injury accounting for 6.8% each; and lumbar three transverse process terminal disease, chronic traumatic synovitis of ankle joint, and bunion at 5.7% [4]. Chan et al. said that the occurrence of trauma is significantly related to excessive specific training, and the athletes' incorrect movement control and fatigue are the key to the occurrence of trauma [5]. Putra et al.'s research found that Chinese elite rhythmic gymnasts have an obvious trend of premature aging caused by sports injuries; especially the younger active athletes have obvious sports injuries [6]. Wilkinson and Mayhew found that the serious injuries of rhythmic gymnasts were in the waist and ankle with the highest incidence rate, moderate injuries have a high incidence of waist, instep, knee, and ankle, and the incidence of minor injuries to the instep, ankle, waist, and shoulder joints is high [7]. In general, the highest incidence of various parts is the waist, followed by the ankle, instep, knee, and shoulder. According to Constantinou et al.'s special survey results, they suggested to arrange training in the basic training stage according to the developmental characteristics of children and adolescents, strengthen the strength training of waist and ankle and other parts, and pay attention to the injury-prone period [8]. Halabchi and Hassabi conducted an injury investigation on 13 national athlete-level and 7 national-level rhythmic gymnasts and found that their injuries were mainly chronic strain injuries of the waist, knees, and feet [9]. The medical supervision of the team found that the main injury of rhythmic gymnasts was vertebral osteomyelitis, after strengthening the strength training of the lumbar and back muscles, and combining with massage, acupuncture, and sealing treatment, symptoms were basically relieved [10]. The results of research on the mechanism of sports injuries in rhythmic gymnasts show that 88.3% had a history of injury. The areas with a higher incidence of injury were the ankle, waist, and knee [11].

## 3. Research Method

### 3.1. Injury Investigation and Analysis of Gymnasts

A survey was conducted on 126 rhythmic gymnasts who participated in the 2011 “Zhongyi Sports Cup” China Rhythmic Gymnastics Championship. The basic situation is shown in Table 1.

A questionnaire survey was conducted on 126 rhythmic gymnastics players who participated in the 2011 “China Art Sports Cup” China Rhythmic Gymnastics Championship, and the results of the survey showed that 98 athletes had injuries of varying degrees, and 28 had no injuries, with a total injury rate of 77.78%, as shown in Table 2.

Through a survey of 126 athletes, the results showed that there were a total of 172 cases (/person) of sports injuries; among the 172 injuries, 30 were acute injuries, accounting for 17.44% of the total injuries. There were 142 chronic injuries, accounting for 82.56% of the total injuries, as shown in Table 3.

Through a survey of 126 athletes, 145 of the 172 injuries were mild injuries, accounting for 84.30% of the total injuries; 25 cases were moderate injury, accounting for 14.53% of the total injury; 2 cases were severe injury, accounting for 1.16% of the total injury, as shown in Table 4.

### 3.2. Overall Incidence of Sports Injuries

As shown in Figure 2, a questionnaire survey was conducted on 126 rhythmic gymnastics players who participated in the 2011 “China Art Sports Cup” China Rhythmic Gymnastics Championship, and 102 athletes had injuries of varying degrees; the survey results showed that there were 172 cases (/person-time) of sports injuries, and the total injury rate was 80.95%. The situation was very serious and posed a great threat to the development of Chinese rhythmic gymnastics. This shows that during the development of rhythmic gymnastics, more attention should be paid to athletes' injuries, and active and effective preventive measures should be taken; avoiding or reducing the occurrence of sports trauma as much as possible has become an important issue to be solved urgently [12].

Through a survey of 126 sports athletes, 32 of the 172 injuries were acute injuries, accounting for 18.60% of the total injuries. There were 140 chronic injuries, accounting for 81.40% of the total injuries. As in most competitive sports, chronic injuries are still common in rhythmic gymnastics, and the proportion is much higher than in other sports [13].

Due to the increased technical difficulty and the increase in exercise training time, load, and density, the incidence of chronic injuries has gradually increased. In addition, if systemic rehabilitation training is not carried out after acute injury, the acute injury will gradually turn into chronic injury [14]. It shows that there are still shortcomings in the current control of chronic injury and the solution of rehabilitation training after injury.

It can be seen from the survey that the sports injuries in rhythmic gymnastics are mainly mild injuries. Moderate and severe injuries force athletes to stop training and rest, which can have a greater impact on training and competition. This prompts us to prevent microduplication and actively take and improve the prevention and rehabilitation measures of injury, so as to reduce the probability of injury.

Among the 172 injuries in this investigation, 0 was skin injury, accounting for 0% of the total injury; 84 cases of skeletal muscle injury, accounting for 48.84% of the total injury; 35 cases of joint injury, accounting for 20.35% of the total injury; and 52 cases of bone injury, accounting for 30.23% of the total injury. There was 1 case of nerve injury, accounting for 0.58% of the total injury [15]. Obviously, skeletal muscle injuries and skeletal injuries account for the majority of sports injuries in rhythmic gymnastics [16]. Skeletal muscle injuries are mainly strains; it shows that the problem of muscle strength and posttraining recovery of rhythmic gymnasts should be highly valued.

### 3.3. Effects of Injury

The reason for the ankle injury is because rhythmic gymnastics is a ballet-based combined equipment (loop, ball, stick, belt, and rope) competitive events, so the movements are mostly done in the state of standing on the heels, and the weight of the human body must be on the ankles. In addition, when jumping, balancing, and rotating, the center of gravity of the human body shifts, and the gravity falls on the outer edge of the foot, causing uneven stress on the ankle and uneven stress between the muscles and ligaments of the ankle; it is easy to cause plantar flexion and varus sprain of the foot, which can damage the lateral synovium of the ankle joint and the anterior talofibular ligament.

Although the athlete had simple strength training, due to the lack of systematic rehabilitation training, it still feels pain; this may also be the main reason why all of his present injuries were to the right extremity. In order to avoid the pain during the movement of the right ankle joint, the movement pattern on the kinematic chain changes, which leads to an increase in the load on other parts, and the long-term accumulation results in the occurrence of injury [17]. Therefore, the pain in this part should be eliminated as soon as possible, and systematic rehabilitation training should be carried out to ensure that it can complete the training task and participate in the competition.

Rhythmic gymnastics requires the conversion of various difficult movements such as jumping, spinning, and rolling in a short period of time; especially in the process of jumping and spinning, due to the instability of the center of gravity, the knee joint often flashes sharply from side to side, and there are flexion, extension, and twisting movements. This can easily cause damage to the medial and lateral meniscus.

The player had obvious pain points in the anterior horn of the lateral meniscus of his right knee, and he had been closed twice because of the pain affecting training, but the effect was not obvious [18]. In the complete set of movements, there are many rotation movements that require the knee joint to be straightened and used as a support; due to the existence of this pain point, players are either unable to complete or are very strenuous, and this can also cause functional compensation of other joints and muscles in the kinematic chain, thereby increasing the risk of injury by overloading these joints. Due to the approaching competition and heavy training tasks, the scientific research team negotiated with leaders, coaches, and players to choose conservative treatment. Therefore, a rehabilitation program was developed for them to ensure that they can train normally and participate in competitions [19].

Precompetition strain on the right waist is an important cause of low back pain, it is very common among athletes, the completion of many movements in rhythmic gymnastics involves flexion and extension of the waist, and the range is large. Therefore, the waist of rhythmic gymnastics athletes needs not only good flexibility but also good core strength.

Many athletes suffer from acute sprained waist without timely treatment and focus on future rehabilitation, resulting in gradual strain [20]. Lumbar muscle strain causes blood circulation disorders and fibrin adhesions can cause pain. Fascial adhesions cause pain, one is the traction of adhesions, and the other is that most of the adhesions have posterior cutaneous branches of spinal nerves, and the adhesion or adhesion of the nerves is involved during exercise, causing pain or numbness. Most patients can still adhere to the training of small and medium amount of exercise, often manifested as pain before and after training [21].

After the athlete suffered an acute back injury, the treatment and rehabilitation were incomplete, and he started training or was gradually strained. In addition, sweating and getting cold during training is also one of the important reasons. When the waist is cold at night, morning stiffness will appear, after warming up, the pain and stiffness disappear, and pain also occurs after a lot of exercise.

According to his symptoms, a set of individualized rehabilitation programs for his waist was formulated to eliminate pain as much as possible, strengthen core strength, and ensure his normal precompetition training and participation in competitions.

Assuming that the lengths of the big arm and the forearm are lu and ll, respectively, we can describe the position of each joint in the SCS coordinate system. Our SCS coordinate system is where the body plane (chest) represents the XZ plane and the body is oriented in the Y direction. The midpoint between the feet is the origin of the SCS coordinate system. Therefore, according to the Denavit-Hartenberg transformation rules, we can calculate the elbow and wrist joints accordingly. For example, when calculating the elbow joint position Pe, we can use the arm length lu to calculate according to the following formula, as shown in

(1) $$\begin{array}{c} \text{Pe}=\text{Ps}+\text{lu}\sin\psi 2, \end{array}$$

(2) $$\begin{array}{c} \text{Pe}=\text{Ps}+\text{lu}\left(\cos\psi 2\times \sin\psi 1\right), \end{array}$$

(3) $$\begin{array}{c} \text{Pe}=\text{Ps}+\text{lu}\left(-\cos\psi 1\times \cos\psi 2\right), \end{array}$$

where Ps is the position of the shoulder joint, and f(∗) calculates the orientation vector from the shoulder joint to the elbow joint. Similarly, the position Pw of the wrist joint can also be calculated accordingly, as shown in

(4) $$\begin{array}{c} \text{Pw}=\text{Pe}+g\left(\psi 1,\psi 2,\psi 3,\psi 4,Ll\right). \end{array}$$

Therefore, according to Equation (1), the phase changes of labels *b* and *r* at these two positions (l0 and ls) can be expressed, as shown in

(5) $$\begin{array}{c} \Delta \theta \left(b,a\right)=\theta \beta \left(b,a\right)-\theta 0\left(b,a\right), \end{array}$$

(6) $$\begin{array}{c} \Delta \theta \left(r,A\right)=\theta \beta \left(r,A\right)-\theta 0\left(r,A\right), \end{array}$$

where |.| is used to calculate the Euclidean distance and *w*(*B*) represents the phase change due to label angular rotation. The phase shift of the tag caused by the hardware can be completely eliminated here. Theoretically, if the distance AO is much larger than the distance |Tb,oO|, then the change of |ATb,p|-|ATb,o| can be approximated as the projection of the distance difference △*x* on the collinear direction, as shown in

(7) $$\begin{array}{c} \Delta xb=\left|Tb,0O\right|\left(1-\cos\beta \right). \end{array}$$

Similarly, we can also calculate the distance difference Δ*xr* of the red label, as shown in

(8) $$\begin{array}{c} \Delta xr=\left|Tr,0O\right|\left(1-\cos\beta \right). \end{array}$$

Therefore, given the distance between labels |*Tb*, *oTr*, *o*|, we can calculate the deflection angle *β* from it.

Through the investigation, it was found that the top three injured parts were the spine, ankles, and lower limbs, which was consistent with the characteristics of rhythmic gymnastics. Rhythmic gymnastics is a skill competition that requires a combination of various complex movements such as balance, jumping, turning, and similar skill movements. The spine is the hub of the trunk activity, and the muscles are the driving force of the spine movement [22]. Injuries to the spine include injuries to the five upper vertebral bodies, muscles, ligaments, and fascia of the cervical, thoracic, lumbar, sacral, and coccygeal vertebrae.

Rhythmic gymnastics requires athletes to have good spine flexibility and strong muscle strength and to establish stable dynamic stereotypes in order to complete difficult and complex movements. Rhythmic gymnastics spine movement range is large, speed is fast, and braking is too much; if the strength is insufficient and the movement is incorrect, it is easy to cause local cumulative damage; the muscles of the spine are rich, different in size, different levels, insufficient, or unbalanced muscle strength, which will cause deformation of the spine, such as cervical vertebral arch and thoracic scoliosis. The survey shows that the spinal curvature of athletes is very obvious, and the degree is different, and the deformation of the spine will in turn affect the center of the entire kinematic chain; then, a vicious circle occurs, which affects the training and competition of the players to a large extent. The injury to the spine greatly exceeds that of the knee and ankle joints in the past, accounting for 39.53% of the total injury; it is suggested here that the prevention and treatment of spinal injury is an urgent problem to be solved.

The spine is the central axis and pillar of the human trunk and has the function of supporting the load, and the spine is an arched structure with good elasticity, which plays the role of transmitting pressure and buffering vibrations [23, 24]. The spine performs various basic movements, acts as a lever for movement, and is the attachment point for many muscles. The characteristics of this project make the development of muscle strength on both sides of the spine unbalanced; as a result, the spine deforms, which in turn leads to a series of skeletal, muscle, and fascia injuries, without systematic rehabilitation training; these injuries lead to a vicious circle, which seriously affects the training and competition of athletes. The muscles on both sides of the spine are very rich, and the balanced development of muscle strength is the key to solving spinal injuries; therefore, attention should be paid to the development of muscle balance in the treatment and rehabilitation of spinal injuries, and strengthen core strength training, thereby reducing spinal deformation, thereby reducing damage to various structures on the spine. First, the weak chain is found through the muscle strength test. While the strength on both sides should be strengthened, the weak side should be developed, but the stretching of the strong side should not be ignored. Deep-level muscle strength should be trained to strengthen the stability of the spine, so that the spine is a normal physiological structure. In the recovery training, therapeutic manipulations, manipulation of spine, application of spinal guns, traction, etc. are added. Treatment and rehabilitation are combined with each other and penetrate each other, so as to achieve the purpose of spinal rehabilitation [25].

The reason for ankle injury is because rhythmic gymnastics is an athletic event based on ballet combined with equipment (rings, balls, sticks, belts, and ropes), so the movements are mostly completed in the state of standing on the heels, and the weight of the human body rests on the ankle [26]. In addition, when jumping, balancing, and rotating, the center of gravity of the human body is offset, and the gravity falls on the outer edge of the foot; uneven force on the ankle and uneven force between the muscles and ligaments of the ankle can easily cause plantar flexion and varus sprain of the foot and damage the lateral synovium of the ankle joint and the anterior talofibular ligament. If there is no systematic rehabilitation training, it is easy to cause repeated ankle injuries [27]. The inherent characteristic of rhythmic gymnastics is the feet walk in a “V” shape, so the outward opening training is an indispensable and important link for rhythmic gymnasts; in addition, the hip joint must be rotated to the maximum extent in the external opening training of the lower limbs, so that the centers of the hip, knee, and ankle joints are always in a straight line. However, if you start a “V” step, you must twist the ankle joint, so that the inner edge of the front foot touches the ground and “falls down”; in this state, the mother toe is in the pronation position, and the ankle joint does not fit in the groove, causing trauma such as ankle synovitis, bunion, and hallux valgus over time. The high incidence of ankle injuries should not be underestimated, as it often affects whether players can train and compete normally. Therefore, foot and ankle injuries should be given full attention, and it is very important to combine treatment with rehabilitation training, especially functional training after ankle injuries. A support belt or brace can be applied to the ankle before training, thereby reducing the occurrence of damage or preventing the recurrence of damage. Timely treatment after injury is the key; RICE, treatment, and rehabilitation after the acute phase cannot be ignored. After an injury, the muscle strength of the ankle joint, the range of motion of the joint, and the tissues around the joint need to be restored. For the complete rehabilitation of the foot and ankle in addition to normalization of its anatomy and tissue, it should also include the recovery of the complex functional capabilities of the site. For the balance function, this ability is extremely important for technologies such as landing buffers. The recovery of functional ability requires the muscles of the ankle to restore the ability to coordinate work and fine work [28].

## 4. Results and Analysis

The 172 cases of injury and illness in this investigation were treated by the following methods: massage, acupuncture, dressing, sealing, strength training, foot soaking, stretching, cupping, ice compress, scraping, repositioning, limbs, acupuncture, immobilization, nutritional medicine, and physiotherapy (mainly medium frequency, ultrashort wave, and roasting electricity). From the above statistics, it can be found that most of the injuries are treated by traditional methods, with acupuncture and massage therapy taking the initiative; the use of taping, ice compress, physiotherapy, rehabilitation training, and other methods still accounts for a small proportion. Most athletes in the survey reported that traditional treatment methods are effective in resolving pain from acute injuries, but injuries tend to recur frequently.

For the complete rehabilitation of the injured part, in addition to the normalization of its anatomical structure and tissue, it should also include the recovery of the complex functional capabilities of the part. The recovery of functional ability requires muscle groups to restore the ability to coordinate work and fine work, and the current injury treatment does not cover the content of rehabilitation training; thorough treatment of the injured area was neglected. In this case, repeated training will cause the injury to accumulate and gradually aggravate into a chronic injury.

The application of necessary support belt fixation technology and protective equipment is important, the application of joint support belt is an important means and effective method to control and protect knee and ankle joint injuries, and the application of knee pads can protect the impact of the carpet on the knee joint. The application of intramuscular effect has a good effect on the prevention of muscle and joint damage. Therefore, it is necessary for us to strengthen the application of taping in rhythmic gymnastics, so as to reduce the occurrence and aggravation of injury.

Strengthen strength training, especially specific muscle strength training, strength training for small muscle groups and core strength training. Core strength training can significantly alter trunk stability in rhythmic gymnasts.

In order to achieve scientific training, on the one hand, we must do a good job of medical supervision: before training, the support belt fixation of vulnerable parts, wearing protective gear and other protective measures, paying attention to the warm-up activities before training, is conducive to reducing the occurrence of injury. After training, athletes can be fully relaxed by various means, especially the athlete's active stretching and relaxation; this can not only fully relax the athlete but also enhance the flexibility of the athlete's whole body, so that the body can more coordinately complete difficult movement techniques. Strengthen the standardization of technical movements during training and treat them differently. Athletes should take effective treatment in time after injury. Another aspect of scientific training is to do a good job of monitoring physiological and biochemical functions and to use scientific means to ensure a reasonable amount of training for athletes.

The best way to recover is to strengthen your core, especially your back. Specifically, training equipment such as elastic bands and Swiss balls is used to exercise, so as to improve the muscle strength of the core and reduce the risk of waist injury.

Increase asymmetrical movement exercises to strengthen stability and agility in asymmetrical states. Pay attention to stretch the tissues around the ankles, knees, and hips to maintain optimal joint mobility.

Strengthen core stability training and improve the stability of limbs and the ability to work together with muscles when supported on one or both sides. Stability exercises can be performed on Swiss balls and balance pads; for example, the single-leg support half squat, the supine, prone, and side-lying static support movements on the Swiss ball can reduce the chance of sports injuries.

## 5. Conclusion

Injury risk assessment provides a theoretical basis for the prevention and rehabilitation of rhythmic gymnasts' injuries; in each stage, an injury risk assessment test is conducted for athletes in the mode of assessment-rehabilitation-reassessment; this guides the implementation of rehabilitation measures at each stage. According to the results of the injury risk assessment, a personalized sports rehabilitation plan is scientifically formulated and implemented, so as to effectively control the injury problem of an athlete and ensure the normal training before the competition, and participated in the 2012 London Olympic Games in the best state, and achieved a historic breakthrough in the performance of China's rhythmic gymnastics individual events. It is proved that through the investigation of 126 rhythmic gymnasts participating in the 2011 “China Art Sports Cup” China Rhythmic Gymnastics Championship, the injury characteristics of gymnasts can be found, and the injury risk assessment can be carried out; it effectively solves the problem of the basis for the rehabilitation and prevention of athletes. It satisfies the needs of the athlete's injury risk assessment test, makes up for the deficiency that the gymnast cannot be assessed for injury, and can improve the recovery efficiency of the athlete after injury.

## Figures and Tables

**Figure 1:** Relationship of risk, risk factor, risk event, and risk loss. Understanding the chain of action of risk is of great significance for dealing with risks.

**Figure 2:** Incidence of rhythmic gymnastics injuries. This is during the development of rhythmic gymnastics.

**Table 1:** Basic information of athletes.

*n* = 126	Age (y)	Height (cm)	Weight (kg)	Years of exercise (y)
Woman	15.24 ± 3.44	161.39 ± 7.58	42.84 ± 6.08	6.56 ± 2.95

**Table 2:** Incidence of sports injuries.

*n* = 126	Number of injuries	No injuries	Total
Woman (*n* = 126)	98	28	126
Percentage (%)	77.78	22.22	100

**Table 3:** The nature of sports injuries in rhythmic gymnastics athletes.

Damage nature	Acute injury	Chronic injury	Total
Visits	30	142	172
Percentage (%)	17.44	82.56	100

**Table 4:** Degree of sports injuries among athletes in rhythmic gymnastics.

Degree of damage	Mild	Moderate	Severe	Total
Visits	145	25	2	172
Percentage (%)	84.30	14.53	1.16	100

## Data Availability

The data used to support the findings of this study are available from the corresponding author upon request.
